This article has been retracted.

# Application and the Effect of the Triple Prerehabilitation Nursing Model in the Perioperative Period of Knee Arthroplasty in Diabetic Patients

**DOI:** 10.1155/2022/1858631

**Published:** 2022-08-12

**Authors:** Sisi Zhao, Lingjun Peng, Tingting Mo, Qianzi Ruan

**Affiliations:** ^1^Orthopedics and Traumatology Ward of Integrated Traditional Chinese and Western Medicine, The First People's Hospital of Wenling, Wenling, Zhejiang 317500, China; ^2^Joint Surgery Ward, The First People's Hospital of Wenling, Wenling, Zhejiang 317500, China

## Abstract

**Objective:**

The aim of the study was to explore the application and the effect of the triple prerehabilitation nursing model in the perioperative period of knee arthroplasty in diabetic patients.

**Methods:**

The prospectively included 60 patients with diabetes who underwent total knee replacement were admitted from August 2021 to April 2022 and were divided into 2 groups according to the (1 : 1) ratio. The control group was mainly given routine nursing care. On the basis of the control group, the observation group received triple prerehabilitation nursing. The postoperative knee flexion, hospital for the special surgery knee score (HSS), the daily living ability (Barthel) score, the modified fall efficacy scale (MFES) score, the recovery of the lower-limb muscle strength, and the incidence of complications were compared between the two groups.

**Results:**

The knee flexion degree and lower-limb muscle recovery of the observation group were better than those of the control group at 3 d, 7 d, and 14 d after operation (*P* < 0.05). The HSS score, Barthel score, and MFES score of the observation group were higher than those of the control group (*P* < 0.05). There was no significant difference in postoperative complications between the two groups (*P* > 0.05).

**Conclusion:**

The triple prerehabilitation nursing care for diabetic patients undergoing total knee replacement can promote the recovery of limb function.

## 1. Introduction

Diabetes has become the third largest threat to health after tumors and cardiovascular and cerebrovascular diseases, with an incidence of more than 170 million worldwide [1]. If diabetes is complicated with knee joint diseases, total knee arthroplasty should be performed as soon as possible, which can effectively improve the functional state of the affected limbs and joints, correct joint deformities, and improve the quality of life. Although the treatment effect is remarkable, due to concurrent diabetes, the postoperative recovery time may be prolonged and the possibility of postoperative complications may even be increased. In this regard, medical staff should pay attention to nursing guidance for patients to improve their prognosis [2]. Although routine nursing can provide high-quality care in the perioperative period, it lacks targeted nursing guidance, especially the overall effect of postoperative rehabilitation is poor [3]. Triple prerehabilitation nursing is a newly proposed nursing strategy in recent years. It can be patient-centered, optimize various detailed nursing care, and better promote postoperative functional recovery of patients. However, it is now commonly used in the fields of thoracic surgery and abdominal surgery [4]. Scholars use triple prerehabilitation nursing in patients with diabetes complicated by knee replacement. Due to the late start, the effect is still in the exploratory stage. Based on this, this article conducts an investigation and further explores the advantages of triple prerehabilitation nursing, in order to provide a basis for the improvement of nursing programs in the future.

## 2. Materials and Methods

### 2.1. Basic Information

From August 2021 to April 2022, 60 patients with diabetes who underwent total knee replacement were prospectively selected as the research subjects. They were divided into the observation group and the control group according to the (1 : 1) ratio. In the observation group, there were 19 males and 11 females, with an average age of (62.38 ± 4.25) years, and random blood glucose of (11.35 ± 2.35) mmol/L; bone and joint classification: 20 cases were grade III and 10 cases were grade IV. In the control group, there were 17 males and 13 females, with an average age of (62.49 ± 4.33) years, and random blood glucose (11.29 ± 2.78) mmol/L; bone and joint classification: 18 cases were grade III and 12 cases were grade IV. There was no statistical difference in sex, age, bone, joint grade, and blood sugar between the two groups (*P* > 0.05). The research complies with the Declaration of Helsinki. Inclusion criteria are as follows: ① patients who meet the diagnostic criteria for diabetes [5]; ② all of them have severe knee osteoarthritis and are in line with the indications for knee replacement [6]; ③ patients who are able to perform bilateral lower extremity exercise training before surgery; ④ those aged ≥18 years old; ⑤ those who signed written informed consent should have no communication or cognitive impairment. Exclusion criteria are as follows: ① patients with diabetic foot with poor blood sugar control; ② those with severe peripheral arterial disease; ③ those with abnormal coagulation function; ④ those with bilateral total knee arthroplasty; ⑤ those with combined neurogenic disease that may affect postoperative joint function recovery.

### 2.2. Methods

The control group was mainly given routine nursing care [7], including (1) preoperative nursing: routine examinations were performed before the operation to control the blood sugar level (give oral hypoglycemic drugs or insulin injections) to lay a good foundation for the success of the operation and inform the patients before the operation. The fasting and water duration should be explained to the patient. (2) Postoperative care: ① blood sugar control: we should pay attention to dietary choices such as reasonably mix protein, fat, sugar, and closely monitor postoperative blood sugar changes. For those with high blood sugar, hypoglycemic treatment should be given on time. ② Complication care: nursing staff closely observe the local skin condition of the incision, whether there is bleeding, exudation, etc., and monitor the change in body temperature, nursing staff closely observe venous return, skin temperature, and swelling of the affected limb, and the patient should be instructed to move the ankle joint as soon as possible to prevent thrombosis. ③ Rehabilitation training: rehabilitation training should be carried out step by step, from passive exercise to active exercise.

On the basis of the control group, the observation group received triple prerehabilitation nursing. (1) Formation of a nursing team: it is formed by nurses specialized in accelerated recovery nursing, specialized nurses in rehabilitation, orthopaedic surgeons, and psychiatrists. The members of the team discuss the nursing plan together, conduct a nursing assessment once a week, and adjust the nursing procedures appropriately according to the patient's recovery. (2) Sports training: ① exercise training: the warm-up exercise includes five parts ankle joint movement, trunk movement, body extension, neck movement, and head movement. a: Head movement: the patient takes a standing position, puts hands on both sides naturally, rotates the head to the left and right sides, and repeats it five times; b: body extension: the patient takes a standing position, puts hands on the waist, with the feet and the shoulder width apart, keeps the center of gravity backwards, tries to lean back as far as possible, and then repeats it several times; c: neck movement: it naturally relaxes the neck, and the patient slowly pushes up the lower jaw with one hand, keeps the back stretched, returns to the position, and repeats it several times; d: ankle joint movement: the patient takes the lying or sitting position, straightens one leg, uses the ankle joint as the fulcrum, flexes the toes, and flex the toes for 10 s each; e: trunk movement: the patient takes the standing position, places the hands on the right and left iliac bones, slightly separates the feet, and slowly tries their best to turn the torso. ② Quadriceps strength exercise: a: knee joint exercise: the patient puts a soft pillow under the ankle joint, ties the muscles on the front of the thigh, straightens the knee joint as much as possible, presses down on the bed hard, continues for 10 s, relaxes for 10 s, and repeats it several times; b: knee extension exercise: the patient ties an elastic motion fixing belt on an immovable object. The patient sits in a chair with armrests and a backrest, ensuring that the edge of the seat is 2 cm behind the knee, and a soft pillow is placed under the thigh. The patient wraps the elastic belt around the ankle, lean backs against the back of the chair, lifts the leg with the fixed belt off the ground, extends the knee joint forward, parallel to the ground, holds the position for 4 seconds, slowly flexes the knee joint until it remains at 80°∼90°, and holds the back position for 4 seconds; c: recumbent straight leg raising training: the patient straightens both lower limbs, raises the legs alternately, leaves the bed at the highest position, holds the position for 10 s, gently lowers it, and repeats it 10 times. ③ Balance exercises include stair climbing, tip-toe walking, heel walking, standing on one leg, sitting and walking on the left and right sides, walking with “8” characters, walking backwards with auxiliary tools, and bending your knees. (3) Nutritional support: we should maintain a balanced choice of food, we should choose appropriate food according to the patient's preference, condition, and taste, we should limit the intake of high-fat and high-calorie diet, change unhealthy eating habits, and appropriately increase high-quality protein (soybeans, eggs, milk, lean meat, and fish) and fresh fruits and vegetables, and we should selectively supplement whey protein powder according to the situation. We should choose the quantitative supplement method, 15 g per day for women and 20 g per day for men, so as to promote muscle synthesis (4) Psychological intervention: during the training period, it is necessary to cooperate with psychological counseling to teach patients some techniques to eliminate anxiety, such as breathing training and relaxation training to relieve inner anxiety, tension, and other emotions.

### 2.3. Observation Indicators

(1) We should instruct the patient to take the supine position, straighten the legs, bend the lower legs, and the fixed arm should be parallel to the longitudinal axis of the femur, and we should use a protractor to align the lateral malleolus of the femur and measure the knee joint before and 3 d, 7 d, and 14 d after the operation. (2) Hospital for the special surgery knee score (HSS) score [8]: 14 days after the operation, we should evaluate the patient's preoperative and postoperative joint stability, flexion deformity, muscle strength, range of motion, limb function, and other items, with a maximum score of 100 points. >85 points are excellent, 70–84 points are good, 60–69 points are fair, and <60 points are poor. The higher the score, the better joint function. Abilities of the daily living (Barthel) score [9]: 14 days after the operation, we should evaluate 10 items such as going up and down stairs, control of bowel and bladder, bathing, eating, and going to the toilet, with a maximum score of 100 points. The better the ability of daily living, the higher the score. The modified fall efficacy scale (MFES) score [10]: 30 days after the operation, 14 items including bathing, changing clothes, getting in and out of bed, simple shopping, and crossing the road should be evaluated, and each item is marked with 0–10 points, if the score is lower, it indicates the greater degree of fear of falling. (3) 30 days after the operation, the recovery of lower extremity muscle strength was recorded: The lower extremity muscle strength was divided into 5 grades according to the examination. Normal muscle strength: Grade 5; limbs can resist partial resistance: Grade 4; the limb cannot resist the resistance, and the limb can be raised: Grade 3; limbs cannot be lifted off the bed surface but can only be moved in parallel on the bed: Grade 2; the limbs cannot complete the movement, only the muscles can contract: Grade 1; complete paralysis: Grade 0. (4) Complications such as lower extremity venous thrombosis, postoperative infection, and prosthesis loosening were compared between the two groups within 30 days after the operation.

### 2.4. Statistical Processing

SPSS 20.0 statistical software was used for processing, and measurement data were represented by ($\bar{x}\pm s$). The differences between the two groups at multiple time points were analyzed by repeated measure analysis of variance. Pairwise comparisons were performed using the LSD-t-test. The count data are expressed in (%), and generalized estimating equation analysis and the *χ*^2^ test were performed. *P* < 0.05 indicated a statistically significant difference.

## 3. Results

### 3.1. Comparison of Knee Flexion Degrees

Repeated measure data analysis of variance showed that knee flexion was statistically significant in terms of the time factor and group interaction (*P* < 0.05). After the pairwise comparison of LSD-t, there was no significant difference in preoperative knee flexion (*P* > 0.05). However, the recovery of knee flexion in the observation group was better at each time period after operation (*P* < 0.05) as shown in Table 1.

### 3.2. Comparison of HSS Scores

The preoperative HSS score of the observation group was (56.65 ± 4.15), and the HSS score was (88.65 ± 2.32) at 14 days after the operation; the preoperative HSS score of the control group was (56.79 ± 4.23), and the HSS score at 14 days after the operation was (81.02 ± 2.41). The postoperative HSS score of the observation group was higher than that of the control group (*t* = 12.837; *P* < 0.001) as shown in Figure 1.

### 3.3. Comparison of Barthel Scores

The Barthel score of the observation group was (62.35 ± 2.32) before the operation, and the Barthel score was (90.68 ± 2.11) at 14 days after the operation; In the control group, the Barthel score was (62.49 ± 2.55) before the operation, and the Barthel score was (82.79 ± 2.52) at 14 days after the operation. The postoperative Barthel score in the observation group was higher than that in the control group (*t* = 13.250; *P* < 0.001) as shown in Figure 2.

### 3.4. Comparison of MFES Scores

The preoperative MFES score of the observation group was (60.87 ± 2.15), and the 30-day postoperative MFES score was (86.65 ± 2.54). In the control group, the preoperative MFES score was (60.59 ± 2.43) and the postoperative 30-day MFES score was (80.32 ± 2.11). The postoperative MFES score of the observation group was higher than that of the control group (*t* = 10.488; *P* < 0.001) as shown in Figure 3.

### 3.5. Comparison of Lower-Limb Muscle Strength Recovery

The recovery of lower-limb muscle strength in the observation group was better than that in the control group (*P* < 0.05) as shown in Table 2.

### 3.6. Comparison of Complication Rates

In the observation group, 1 case of infection and 1 case of lower extremity venous thrombosis occurred after the operation, totaling 6.67% (2/30). In the control group, there was 1 case of prosthesis loosening, 1 case of postoperative infection, and 1 case of lower extremity venous thrombosis, totaling 10.00% (3/30). There was no significant difference in postoperative complications between the two groups (*χ*^2^ = 0.218; *P*=0.640) as shown in Figure 4.

## 4. Discussion

With the improvement of the application of imaging technology and computer simulation technology, total knee arthroplasty has been promoted in clinical practice. Compared with traditional surgical methods, it is more in line with the biomechanical characteristics of the knee joint, can improve the function of the knee joint, relieve local pain, and improve the quality of life. Total knee arthroplasty has irreplaceable advantages, but for patients with concurrent diabetes, it can increase the risk factor of surgery, cause a stress response, and affect the prognosis. For this, corresponding nursing guidance should be given according to the characteristics of the patient's condition to improve the prognosis [11, 12]. In the past, it was difficult for routine nursing to meet the needs of such special groups of patients. It is necessary to provide patients with more satisfactory, more complete, and more comprehensive nursing services through innovative nursing models so as to ensure the quality of nursing and to meet the needs of patients [13]. With the promotion of the concept of fast recovery, scholars have found that it can greatly improve the prognosis and promote postoperative recovery [14]. The triple prerehabilitation nursing is a comprehensive nursing plan based on the concept of rapid rehabilitation. The nursing mode is divided into three aspects, namely, rehabilitation nursing, nutritional support, and psychological support. It can better promote the patient's recovery after surgery, but there are few relevant studies in my country, and the effect remains to be explored.

Analysis of the results of this study showed that there was no statistical difference in postoperative complications between the two groups, indicating that paying attention to preoperative and postoperative nursing in routine nursing can lay a good foundation for postoperative rehabilitation and prevent postoperative complications. In addition, compared with the control group, the observation group had better knee flexion, lower-limb muscle strength recovery, and higher HSS score, indicating that triple prerehabilitation nursing can better prevent muscle atrophy around the knee joint, give full play to “brain plasticity”, and increase muscle strength. Triple prerehabilitation nursing can fully mobilize various reflexes of the body, better restore the maximum muscle strength of the limbs, and improve the function of the limbs. We analyze the reasons as follows: on the one hand, triple prerehabilitation nursing fully considers the anatomical position and stress of the knee joint and adopts a special biomechanical movement mode, such as ankle joint, trunk, neck, head movement, and body extension, which is beneficial to the recovery of the quadriceps femoris muscle and prevent knee flexion contracture [15]. On the other hand, early standardized exercise can prevent joint capsule and tendon contractures and adhesions, enhance muscle strength, increase local blood circulation, soften scars, improve knee joint function, and restore normal limb and joint function [16, 17]. In addition, the Barthel score and MFES score of the observation group were higher than those of the control group. This shows that triple prerehabilitation nursing can better improve the patients' cooperation, enthusiasm, and initiative, promote disease recovery, and improve the quality of life. In triple pre-rehabilitation nursing, warm-up exercise, balance training, and quadriceps strength exercise can improve the swelling of the surgical site, promote venous lymphatic return, prevent the occurrence of flexion contracture, improve the function of the knee joint and the contraction ability of the surrounding muscles, enhance the strength of the knee joint, and improve the postoperative quality of life. Through nutritional support, the body's nutrient needs can be supplemented and the body's resistance and immunity can be improved. Psychological intervention can stabilize patients' emotions so that rehabilitation training can be carried out smoothly [18, 19].

In conclusion, triple prerehabilitation nursing can promote functional rehabilitation of the knee joint and improve postoperative discomfort symptoms. However, this study also has shortcomings. First, the sample size is limited, and second, long-term follow-up and observation are not carried out. Therefore, the long-term effect of this nursing model remains to be explored.

## Figures and Tables

**Figure 1:** Comparison of the HSS scores between the two groups.

**Figure 2:** Comparison of the HSS scores between the two groups.

**Figure 3:** Comparison of the MFES scores between the two groups.

**Figure 4:** Comparison of complications between the two groups.

**Table 1:** Comparison of knee flexion degrees between the two groups at different time periods.

Group	*n*	Preoperative	3 d after surgery	7 days after surgery	14 days after surgery
Observation group	30	77.46 ± 4.52	88.61 ± 5.32	94.78 ± 5.54	104.68 ± 7.19
Control group	30	77.59 ± 4.36	83.33 ± 4.47	89.45 ± 4.39	96.65 ± 6.65
*F* value	—	*F*_time_ = 1675.532, *F*_Interaction_ = 44.532, *F*_betweenthegroups_ = 15.419			
*P* value	—	*P* time < 0.001, *P* Interaction < 0.001, *P* between the groups < 0.001			

**Table 2:** Comparison of the recovery of lower-limb muscle strength between the two groups.

Group	*n*	Grade 0	Grade 1	Grade 2	Grade 3	Grade 4	Grade 5
Observation group	30	0	0	0	1	2	27
Control group	30	0	0	1	2	4	23
*Z* value	—	−5.838					
*P* value	—	<0.001					

## Data Availability

The data used and/or analyzed during the current study are available from the corresponding author on request.
